The article "Performance Evaluation of Bio Concrete by Cluster and Regression Analysis for Environment Protection" was published in 2022. Journal: Comput Intell Neurosci.

# Performance Evaluation of Bio Concrete by Cluster and Regression Analysis for Environment Protection

**DOI:** 10.1155/2022/4411876

**Published:** 2022-09-01

**Authors:** Ashish Shukla, Nakul Gupta, Kunwar Raghvendra Singh, Pawan Kumar Verma, Mohit Bajaj, Arfat Ahmad Khan, Frie Ayalew

**Affiliations:** ^1^Department of Civil Engineering, GLA University, Mathura, Uttar Pradesh 281406, India; ^2^Department of Computer Science Engineering, MIT Art, Design and Technology University, Pune, Maharashtra 412201, India; ^3^Department of Electrical Engineering, Graphic Era (Deemed to Be University), Dehradun 248002, India; ^4^Department of Electrical and Electronics Engineering, National Institute of Technology, Delhi 110040, India; ^5^College of Computing, Khon Kaen University, Khon Kaen 40000, Thailand; ^6^College of Electrical and Mechanical Engineering, Addis Ababa Science and Technology University, Addis Ababa 16417, Ethiopia

## Abstract

The focus of this research is to isolating and identifying bacteria that produce calcite precipitate, as well as determining whether or not these bacteria are suitable for incorporation into concrete in order to enhance the material's strength and make the environment protection better. In order to survive the high “potential of hydrogen” of concrete, microbes that are going to be added to concrete need to be able to withstand alkali, and they also need to be able to develop endospores so that they can survive the mechanical forces that are going to be put on the concrete while it is being mixed. In order to precipitate CaCO_3_ in the form of calcite, they need to have a strong urease activity. Both Bacillus sphaericus and the Streptococcus aureus bacterial strains were evaluated for their ability to precipitate calcium carbonate (CaCO_3_). These strains were obtained from the Department of Biotechnology at GLA University in Mathura. This research aims to solve the issue of augmenting the tension and compression strengths of concrete by investigating possible solutions for environmentally friendly concrete. The sterile cultures of the microorganisms were mixed with water, which was one of the components of the concrete mixture, along with the nutrients in the appropriate proportions. After that, the blocks were molded, and then pond-cured for 7, 28, 56, 90, 120, 180, 270, and 365 days, respectively, before being evaluated for compressibility and tensile strength. An investigation into the effect that bacteria have on compression strength was carried out, and the outcomes of the tests showed that bacterial concrete specimens exhibited an increase in mechanical strength. When compared to regular concrete, the results showed a maximum increase of 16 percent in compressive strength and a maximum increase of 12 percent in split tensile strength. This study also found that both bacterial concrete containing 106, 107, and 108 cfu/ml concentrations made from Bacillus sphaericus and Streptococcus aureus bacteria gave better results than normal concrete. Both cluster analysis (CA) and regression analysis (RA) were utilized in this research project in order to measure and analyze mechanical strength.

The article "Performance Evaluation of Bio Concrete by Cluster and Regression Analysis for Environment Protection" was published in 2022. Journal: Comput Intell Neurosci.

## 1. Introduction

Concrete is thought of as a homogeneous substance since it is created by combining cement, coarse and fine aggregate, and water in a certain ratio. Concrete is a porous material and is sensitive to various assaults such as chloride, CO_2_, sulfate, freeze and thaw cycles, and others because it is made up of voids that are referred to as pores [1, 2]. Since these pores are typically associated with one other, concrete is a porous substance. Concrete has a design life of fifty years, but owing to these assaults, it deteriorates considerably more quickly than expected. The infrastructure is built of concrete [3–5]. Cementitious concrete is the most often used building material and is also one of the most essential substances used in construction business. Its annual production is around 10 km^3^/per year, and it is one of the very important materials in the construction industry. Cement is the sole component that is made, whereas the rest are naturally occurring and sourced from the area [6]. The manufacturing of 1 ton of cement results in the release of around 1 ton of carbon dioxide, and the building industry is responsible for approximately fifty percent of the world's total CO_2_ emissions. Because of its adaptability, concrete is employed in the construction of a wide variety of structures, including bridges, large buildings, off-shore constructions, airports, sidewalks, railroad beds, and deep foundations, despite the fact that it is fragile and has a low resistance to stress [7–9]. A great number of concrete buildings are plagued by early deterioration issues such as carbonation and chloride attack, both of which ultimately result in the buildings needing to be repaired and retrofitted. Over the last several years, research into microbial (CaCO_3_) calcium carbonate has been more popular in the field of building engineering. It is seen as a potentially fruitful novel method for extending the useful life of cement-based buildings [10–12]. The CaCO_3_ calcium carbonate precipitation that results from metabolic activity of various microbe species, such as sulfate-reducing microbes, ureolytic microbes, nitrate reducing microbes, and oxidation of organic microbes, is what allows this method to self-heal the gaps in the concrete and the inevitable microcracks that will form in the concrete. For instance, ureolytic microbes are responsible for the production of an enzyme known as urease, which decomposes urea into carbonate ions [13, 14]. According to the findings of our earlier studies, the process of carbonate precipitation by microbes was carried out by utilizing ureolytic microbes. Since they produce an enzyme called urease, these microbes are able to affect the precipitation of CaCO_3_ in a given environment. This enzyme catalyzes the hydrolysis of urea into carbon dioxide and ammonia, which ultimately results in a rise in both the pH and the amount of carbonate in the surrounding/environment in which the microbes are found. The incorporation of microbial species into concrete has increased its strength and endurance, providing additional benefits in the form of environmentally friendly and cost-effective alternatives. Since bacteria thrive at alkaline pH, the concrete's resistance to alkali assault, chemical attacks, freeze-thaw strike, and drying shrinkage is significantly improved [15–17]. In a similar vein, the compression strength of Bio-Concrete was the subject of a great deal of research in order to evaluate the efficacy of bacteria-based self-healing in the existing body of scholarly work. This is due to the fact that the strength of concrete is regarded as an essential metric that represents the uniformity of a concrete mix as well as the components of the material being used [18–20]. The compressive strength test has a direct bearing on the general performance of the concrete as well as its attributes. As a result, the compression strength technique has been widely utilized to analyze the process of microbes-based self-healing in cementitious concrete, combining bacteria and associated chemical compounds in the research that has been published [21, 22]. An examination of the relevant literature reveals that virtually all bacteria are capable of producing calcium carbonate (CaCO_3_) as a precipitate; however, for the selected bacteria to provide the greatest advantages, they must be alkaliphilic and thermophilic. *Bacillus sphaericus*, which is an alkaliphile and precipitates (CaCO_3_) calcium carbonate with a higher density, and *Streptococcus aureus*, which is also an alkaliphile and increases the compressive strength of concrete, are both beneficial microorganisms [23, 24]. For instance, the research group “Chattopadhyay et al.” found that the compression strength of bacterial mortar increased with time, specifically at seven, twenty-eight, and fifty-six days, in comparison to the normal mix. The precipitation of CaCO_3_, which filled the gaps and improved the texture of the concrete as a result, was thought to be responsible for the increase in compression strength that was observed. Additionally, “Ryu et al.” came to the conclusion that the highest increase in compression strength was observed at a microbial cell concentration of 30 × 105 cfu/mL, and also that the compressive strength declined once this value was exceeded [25]. In a similar vein, the “Manikandan et al.” study indicated that a rise in compressive strength occurred even at a high concentration level of 108 cells/mL. In the same vein, the greatest notable improvement in compression strength was seen when there were 10^6^ cells per milliliter of solution [26]. Predictions of compressive strength are extremely valuable because of the significant savings in both money and time that they provide. Because of this fact, researchers have been motivated to construct a mathematical model that correctly forecasts the strength of various forms of concrete. Despite this, there still is not a prediction formula or code requirements for estimating the strength properties of microorganism concrete [27, 28].

The article "Performance Evaluation of Bio Concrete by Cluster and Regression Analysis for Environment Protection" was published in 2022. Journal: Comput Intell Neurosci.

In order to find a solution to the problem of increasing the tensile and compression strengths of concrete, the purpose of this study is to investigate potential options. Microorganisms grown in sterilized cultures were combined with water, which was one of the components of the concrete mixture, along with the nutrients in the right amounts. After that, the blocks were cast, and then they were pond-cured for 7, 28, 56, 90, 120, 180, 270, and 365 days, respectively, before being assessed for compressibility and tensile strength. In order to assess and investigate the nature of mechanical strength, this research study made use of both cluster analysis (CA) and regression analysis (RA). After a thorough study of old papers, the researcher found that not much research has been done with Bacillus sphaericus and Streptococcus aureus bacteria and also found that till date no researcher has done a thorough study of the results through cluster analysis for Bacillus sphaericus and Streptococcus aureus bacterial concrete. The researcher used three different concentrations, namely 106, 107, and 108 cfu/ml, of Bacillus sphaericus and Streptococcus aureus bacteria to determine the relationship between bacterial concrete and normal concrete.

This paper shows the introduction of the study in Section 1 and the materials used for the research in Section 2, bacteria (Bacillus sphaericus and Streptococcus aureus) used in Section 2.1, and research methodology in Section 3.1; Section 3.2 shows bacterial culture techniques, Section 3.3 shows concrete mix design, Section 4 shows results and discussion, and Section 5 shows conclusions.

The article "Performance Evaluation of Bio Concrete by Cluster and Regression Analysis for Environment Protection" was published in 2022. Journal: Comput Intell Neurosci.

## 2. Materials Used

OPC (ordinary Portland cement) of the grade 43 was utilized in this experimental endeavor. In accordance with IS 4031-1996 [29], this OPC was evaluated for both its physical qualities and its optical properties. The specific gravity, Blaine's fineness [30], soundness, and compressive strength of Portland cement were all measured and analyzed to identify their respective qualities [31, 32]. In this particular project, the fine aggregates consisted of river and crushed stone sand, both of which were sourced locally and were readily accessible. Sand from rivers typically has a specific gravity of about 2.68. As a coarse aggregate for this project, crushed granite-shattered stone with a nominal size of 20 millimeters is being employed [33–35]. In the experimental study, safe and potable water that was readily available in the local area was utilized for all combinations.  Table 1 presents the variables studied and the procedure of bacterial concrete.

### 2.1. Bacillus sphaericus Bacteria and Streptococcus aureus Bacteria

Both Bacillus sphaericus and Streptococcus aureus were obtained from the Department of Biotechnology at GLA University in Mathura. The fact that the microorganisms Bacillus sphaericus and Streptococcus aureus are able to survive in the highly alkaline surroundings of concrete during the formation of CaCO_3_ crystals on concrete suggests that the presence of the microbes had no negative implication on the hydration of reaction, which forms a dense CaCO_3_ crystal in liquid medium [39, 61]. Ureolytic, Gram +ve, anaerobic, and round-spore-forming Bacillus sphaericus and Streptococcus aureus at a temperature of four degrees Celsius were grown on nutrient agar slants, and they were subcultured once every fifteen days on a medium that had been filtered and sterilized [59, 62].

## 3. Methodology

### 3.1. Research Methodology

The gathering of particular experimental data that contributes to a better understanding of microorganism concrete and the features it possesses is the primary aim of the current experimental research (durability and strength). In the current experimental inquiry, tests on the behavior of hardened and fresh characteristics of ordinary concrete grade and normal grade concrete without and with the inclusion of microbes have been carried out. These studies were carried out as part of the experimental study. Concrete in its hardened state is subjected to the appropriate laboratory tests, which enable the concrete strength, such as compression strength and tension strength. Research process methodology is shown in Figure 1.

The article "Performance Evaluation of Bio Concrete by Cluster and Regression Analysis for Environment Protection" was published in 2022. Journal: Comput Intell Neurosci.

The primary purpose of this experimental inquiry is to investigate the strength of normal concrete and bacterial concrete. The current work may be broken down into three distinct stages:

  Phase 1: growth of bacteria and culturing technique of bacterial concrete
  Phase 2: to study the compression strength and split tensile strength of bacterial concrete
  Phase 3: regression analysis and cluster analysis

### 3.2. Culturing Technique of Bacteria

Both Bacillus sphaericus and Streptococcus aureus were cultivated in a medium that was designed for the improved generation of CaCO_3_. This medium includes baking soda, ammonium chloride, urea, and CaCl_2_, and it was dissolved in distilled water [36]. In order to determine the growth curve, the colonies were cultivated in batch culture aerobic endurance at 37 degrees Celsius and 100 revolutions per minute for a period of time [37, 41]. During this process, aliquots of the cells were taken out for optical density measurements and standard plate enumeration. We used a UV-vis 3000plus dbl spectrometer [63] to determine the initial concentration at 600 nm, also known as OD 600 (Department of Biotechnology, GLA University, Mathura).

### 3.3. Mix Design of Concrete

Concrete of the grade M30 was mixed in accordance with the standards set out in IS 10262-1982 [64]. For an exposure level of moderate and a water to cement ratio of 0.46, the amount of cement necessary to produce 1 m^3^ of concrete is 400 kg. Casting concrete into cubes of size 100 millimeters by 100 millimeters by 100 millimeters is carried out to determine the concrete's compressive strength, and casting concrete into cylinders of size 100 millimeters in diameter and 200 millimeters in length is carried out to determine the concrete's split tensile strength. Mix design is shown in Table 2.

## 4. Result and Discussion

### 4.1. Compression Strength

The evaluation of the effect that the incorporation of microorganisms into the mixture has on the compression strength and stiffness of cement concrete blocks is another factor that is taken into consideration [65–67]. The compression strength of the concrete was enhanced as a result of the influence of the bacterial isolates, as can be seen in Figures 2, 3, and Table 3. It is clear that the compression strength of microorganism concrete is significantly higher than that of the conventional concrete. The increase in compressive strength that is brought about by bacteria is presumably brought about by the deposition of calcium carbonate [67] on the surfaces of the microbe cell and the gaps inside the concrete, which plugs the holes that are present in the binder matrix [68, 69]. The filling of the gaps inside the concrete with microbiologically generated concrete mixes is the primary cause of the increase in compression strength [70]. The findings of the study indicated that the addition of bacteria to concrete led to an increase in compressive strength, which, in turn, would lead to an improvement in the concrete's overall performance.

The article "Performance Evaluation of Bio Concrete by Cluster and Regression Analysis for Environment Protection" was published in 2022. Journal: Comput Intell Neurosci.

### 4.2. Split Tensile Strength

In order to evaluate the tension strength of each mixture, three cylinders measuring 100 mm by 200 mm were casted for every combination. In order to create these cylinders, a mold made of cast iron and steel was utilized. Casting and curing times for each mix percentage were as follows: seven days, twenty-eight days, fifty-six days, ninety days, one hundred eighty days, two hundred seventy days, and three hundred sixty-five days. In accordance with the Indian Standard code IS 516–1959 [71], a split tensile strength test is performed at the ages of seven days, twenty-eight days, fifty-six days, ninety days, one hundred twenty days, one hundred eighty days, two hundred seventy days, and three hundred sixty-five days using a compressive testing machine with a capacity of two thousand kilonewtons. The loading part and the surface of the cylinder specimen are separated by a wooden strip so that there is no direct impact from the loading on the cylinder [55, 72, 73]. As shown in Figures 4, 5, and Table 4, the effect of the bacterial isolates resulted in an increase in the split tension strength of the concrete. This improvement can be attributed to the fact that the concrete was allowed to cure at a higher temperature [58]. It would suggest that the addition of Bacillus sphaericus and Streptococcus aureus was responsible for the rise in the splitting tension strength.

### 4.3. Predicted Split Tension Strength

The findings of the experiments were evaluated using regression analysis [43], which led to the discovery of the link between the compression strength of microbiological and normal concrete as well as tension strength of microbiological and normal concrete. This relationship may be expressed as equation (1), [74]. The predicted tensile strength's results at different day intervals are shown in Table 5 and Figures 6 and 7.

(1) $$\begin{array}{c} F_{\text{tensile}}=0.23f_{{\text{compression}}^{0.73}}. \end{array}$$

### 4.4. Regression Analysis

The results of an experiment are depicted in Figure 8, which shows the link between the tension strength and the compression strength of bacterial concrete that was made with the bacteria Bacillus sphaericus and Streptococcus aureus. The linear equation displays not only the percentage correlations between compression strength and split tensile strength (*σ*) [75] but also the regression coefficients (*R*^2^) [76] that were derived from the equation that was shown below.

(2) $$\begin{array}{c} y=0.249_{x}-4.4595. \end{array}$$

The following value for the regression coefficient, *R*^2^ (0.8813), indicates that the regression line as well as the statistics of compression strength and split tensile strength values has a solid connection with one another. As can be seen from equation (2), the tensile strength improves as the compressive strength does.

The article "Performance Evaluation of Bio Concrete by Cluster and Regression Analysis for Environment Protection" was published in 2022. Journal: Comput Intell Neurosci.

### 4.5. Cluster Analysis

Multivariate statistical techniques are typically utilized for the categorization, analysis, and interpreting of big data sets. These approaches are also employed for the decrease of a dimension of complicated datasets with a minimal loss of original data [77]. Cluster analysis is a method of unsupervised pattern classification that organizes the objects into the categories (clusters) on the basis of their commonalities within a category and their differences from other categories. The findings of CA lend a hand in data interpretation and point to patterns in the data. The square root of the average squared of the distinctions among corresponding values is computed in order to derive the distance from site in the Euclidean distance, which is one of the measurements that is utilized most frequently in order to determine the degree to which two cases are comparable to one another.

Through cluster analysis, it was found that the compression strength of bacterial concrete SP1, SA 1, SP 2, and SA 2 increases in the same way, and similarly, compression strength of SP3 and SA3 increases in the same group. Also, the compression strength of normal concrete sets itself apart from bacterial concrete. Cluster analysis results for compression strength are displayed in Figure 9.

Through cluster analysis, it was found that the tension strength of bacterial concrete SP 3, SA3, and SA1 increases in the same way, and tensile strength of SP 1, SA2, and SP 2 increases in the same group. Also, the split tensile strength of normal concrete sets itself apart from bacterial concrete. Cluster analysis results for split tensile strength are displayed in Figure 10.

## 5. Conclusion

- The study of this research work has shown that the mechanical strength of concrete can be increased by using Bacillus sphaericus and Streptococcus aureus bacteria for bio-concrete.
- Using both bacteria in concrete with different concentrations showed that microbial concrete with a concentration of 10^7^ cfu/ml produced better results for mechanical strength.
- This study also found that both bacterial concrete containing 10^6^, 10^7^, and 10^8^ cfu/ml concentrations made from Bacillus sphaericus and Streptococcus aureus bacteria gave better results than normal concrete.
- Value of the regression coefficient indicates that the regression line as well as the statistics of compression strength and split tensile strength values has a solid connection with one another.
- Through cluster analysis, it was found that the compression strength of bacterial concrete SP1 and SA1 increases almost equally, similarly, the compression strength of bacterial concrete SP2 and SA2 increases almost equally, and both the compressive strength of both SP3 and SA increases almost equally in a similar group. And in the cluster analysis for split tensile strength, three groups were formed, in which in the first group the tensile strength of SP3, SA3, and SA1 increases almost equally, and in the second group the tensile strength of SP1, SA2, and SP2 is mutual, which grows almost evenly, and in the third group comes the normal concrete.
- Research organizations from all over the worldwide have been interested in the employment of microbes for the purpose of increasing the longevity of construction materials as a consequence of the encouraging findings obtained so far. Our grasp of the opportunities and constraints presented by biotechnological processes on construction materials may unquestionably benefit from the work that has been carried out by a number of research groups that have concentrated their attention on a variety of materials. Studies are still being conducted on the preservation of nutrients and microbial products since these factors have an effect on the survival, development, and creation of biofilms. “Bacillus sphaericus and Streptococcus aureus bacterial concrete” appears to become the most viable technique for generating crack-resistant concrete in the coming days, according to the findings of this research as well as the prior research that has been conducted.

The article "Performance Evaluation of Bio Concrete by Cluster and Regression Analysis for Environment Protection" was published in 2022. Journal: Comput Intell Neurosci.

## Figures and Tables

**Figure 1:** Research process methodology.

**Figure 2:** Graphical representation of compression strength result at different days' intervals.

**Figure 3:** Graphical representation of average compression strength result at different days' intervals.

**Figure 4:** Graphical representation of split tension strength result at different days' intervals.

**Figure 5:** Graphical representation of average split tension strength result at different days' intervals.

**Figure 6:** Graphical representation of predicted split tension strength result at different days' intervals.

**Figure 7:** Graphical representation of average predicted split tension strength result at different days' intervals.

**Figure 8:** Linear regression analysis between compressive and tensile strength.

**Figure 9:** Cluster analysis result of compressive strength.

**Figure 10:** Cluster analysis result of split tensile strength.

**Table 1:** Variables studied and procedures of bacterial concrete.

Materials used	Durability and mechanical test	Existing structure
Pseudomonas bacteria [36–39]	Compression strength [40–42]	Self-healing [16, 43–45]
Bacillus subtilis [2, 4, 34]	Tension strength [5, 46–48]	Resettlement of original structure [1, 16, 49, 50]
Megaterium bacteria [5, 51, 52]	Flexural strength [3], [28, 53, 54]	
Cereus and sphaericus bacteria [55–57]	Durability characteristics [12, 19, 58–60]	

**Table 2:** Materials utilized in concrete mix design in detail.

Concrete	Mix Id	Sample	Bacteria cell concentration (ml)	OPC	Coarse aggregate	Fine aggregate	Water
Normal concrete	Conv.	A	—	400	1457	940	168
		B	—	400	1457	940	168
		C	—	400	1457	940	168

Bacillus sphaericus bacterial concrete	SP1	A	SP10^6^	400	1457	940	168
		B	SP10^7^	400	1457	940	168
		C	SP10^8^	400	1457	940	168
	SP2	A	SP10^6^	400	1457	940	168
		B	SP10^7^	400	1457	940	168
		C	SP10^8^	400	1457	940	168
	SP3	A	SP10^6^	400	1457	940	168
		B	SP10^7^	400	1457	940	168
		C	SP10^8^	400	1457	940	168

Streptococcus aureus bacterial concrete	SA1	A	SA10^6^	400	1457	940	168
		B	SA10^7^	400	1457	940	168
		C	SA10^8^	400	1457	940	168
	SA2	A	SA10^6^	400	1457	940	168
		B	SA10^7^	400	1457	940	168
		C	SA10^8^	400	1457	940	168
	SA3	A	SA10^6^	400	1457	940	168
		B	SA10^7^	400	1457	940	168
		C	SA10^8^	400	1457	940	168

**Table 3:** Compression strength result at different days' intervals.

Day	Sample	Normal concrete	Bacillus sphaericus bacterial concrete			Streptococcus aureus bacterial concrete		
			10^6^ cfu/ml	10^7^ cfu/ml	10^8^ cfu/ml	10^6^ cfu/ml	10^7^ cfu/ml	10^8^ cfu/ml
7 days	A	21.71	26.32	27.31	25.53	24.91	25.61	23.36
	B	20.39	25.16	26.63	25.32	23.31	25.74	22.34
	C	19.86	25.72	27.81	26.72	23.67	23.31	23.91

28 days	A	35.61	39.72	40.19	38.32	38.61	39.65	37.31
	B	36.32	38.31	41.62	39.61	38.39	38.23	35.64
	C	35.68	37.69	40.03	38.59	37.42	39.69	37.65

56 days	A	40.88	42.39	44.39	41.67	43.23	45.37	42.37
	B	40.32	40.61	43.27	40.31	42.64	44.47	41.86
	C	41.23	42.13	43.53	40.63	41.35	44.83	43.73

90 days	A	43.61	49.24	49.57	47.67	49.23	49.91	47.21
	B	41.08	49.67	47.62	45.34	48.27	48.07	46.63
	C	42.71	48.63	49.67	47.57	49.86	49.03	47.67

120 days	A	45.83	51.71	52.37	49.54	52.71	53.43	49.87
	B	44.65	52.16	50.33	48.62	52.65	53.41	49.31
	C	45.79	51.75	52.64	49.37	53.53	52.62	49.64

180 days	A	47.64	53.62	54.45	51.47	54.43	55.53	51.07
	B	47.64	53.49	53.43	50.39	53.41	55.61	52.31
	C	46.59	51.35	53.06	50.87	53.63	55.39	50.03

270 days	A	46.23	55.12	56.39	52.39	56.86	57.74	52.75
	B	48.23	53.19	54.71	52.61	55.37	56.81	51.21
	C	48.17	55.64	56.23	52.39	56.26	56.37	52.86

365 days	A	49.13	56.87	57.61	53.67	56.07	58.96	53.39
	B	49.08	56.61	56.63	54.89	56.61	57.07	53.61
	C	50.23	56.12	57.81	52.93	57.37	58.83	53.37

The article "Performance Evaluation of Bio Concrete by Cluster and Regression Analysis for Environment Protection" was published in 2022. Journal: Comput Intell Neurosci.

**Table 4:** Tension strength result at different days' intervals.

Day	Sample	Normal concrete	Bacillus sphaericus bacterial concrete			Streptococcus aureus bacterial concrete		
			10^6^ cfu/ml	10^7^ cfu/ml	10^8^ cfu/ml	10^6^ cfu/ml	10^7^ cfu/ml	10^8^ cfu/ml
7 days	A	2.03	2.68	2.91	2.39	2.31	2.56	2.3
	B	2.11	2.39	2.89	2.41	2.29	2.63	2.16
	C	2.13	2.7	2.93	2.52	2.17	2.81	2.21

28 days	A	3.16	4.51	5.31	4.31	4.62	6.02	4.27
	B	3.23	4.31	5.62	4.16	3.98	6.13	4.31
	C	3.68	5.03	5.17	4.39	4.57	5.87	3.92

56 days	A	4.16	6.23	7.08	5.23	5.17	6.31	5.13
	B	4.39	6.13	7.16	5.16	5.93	6.42	5.31
	C	4.08	6.27	7.11	5.39	5.23	5.98	5.27

90 days	A	5.09	7.18	8.21	6.08	6.14	7.21	6.17
	B	5.67	7.23	8.18	6.17	6.31	7.52	6.19
	C	5.83	6.98	8.31	5.87	5.93	7.43	6.45

120 days	A	5.98	8.17	9.17	7.17	8.03	8.13	7.17
	B	5.87	8.31	9.19	7.77	8.12	8.39	7.13
	C	5.92	8.42	8.92	7.52	8.11	7.81	7.06

180 day's	A	6.13	9.16	10.16	8.13	8.87	9.16	8.16
	B	6.34	9.38	10.23	8.91	8.92	9.23	8.32
	C	6.24	8.93	10.08	7.86	8.99	9.33	8.05

270 days	A	6.87	10.19	11.26	8.17	9.62	10.19	8.91
	B	6.67	9.89	11.38	8.39	9.39	10.27	8.89
	C	6.54	10.21	10.97	8.17	8.91	9.89	7.98

365 days	A	6.91	11.31	12.03	9.16	10.11	11.61	9.17
	B	6.97	11.22	11.98	9.71	10.27	11.91	9.23
	C	7.08	11.34	11.91	8.98	10.33	11.89	9.31

**Table 5:** Predicted tensile strength result at different days' intervals.

Day	Sample	Normal concrete	Bacillus sphaericus bacterial concrete			Streptococcus aureus bacterial concrete		
			10^6^ cfu/ml	10^7^ cfu/ml	10^8^ cfu/ml	10^6^ cfu/ml	10^7^ cfu/ml	10^8^ cfu/ml
7 days	A	2.038227629	2.503436224	2.571832482	2.448358056	2.404809379	2.453956321	2.294631801
	B	2.077793632	2.422404145	2.524926774	2.433640017	2.291045402	2.463043444	2.221051093
	C	2.038227629	2.461646233	2.606120893	2.531153289	2.316821444	2.291045402	2.333946661

28 days	A	3.121586521	3.380684022	3.409839839	3.293278443	3.31145373	3.376333718	3.229685754
	B	3.166899629	3.292651047	3.497988291	3.373846899	3.297668971	3.287630294	3.123506065
	C	3.126064779	3.253665605	3.399924843	3.310201448	3.236634043	3.37881986	3.251144495

56 days	A	3.452476917	3.545113386	3.6664519	3.501055467	3.596259797	3.725366843	3.543892297
	B	3.417887928	3.435816163	3.598688612	3.417269093	3.560363902	3.671274354	3.512701689
	C	3.474030048	3.529227066	3.614461166	3.437051316	3.481408306	3.692946494	3.626576596

90 days	A	3.619309138	3.954758866	3.97408953	3.862307051	3.954172543	3.993969665	3.835064357
	B	3.464799065	3.979940439	3.859349338	3.723568456	3.897734599	3.885938698	3.800612473
	C	3.564629716	3.91893403	3.979940439	3.856390786	3.991048415	3.942439324	3.862307051

120 days	A	3.752902069	4.098616165	4.136738945	3.972333635	4.156327281	4.197696287	3.991632728
	B	3.682116322	4.124623116	4.018477076	3.918345731	4.152873001	4.196549189	3.958862225
	C	3.750510674	4.100930361	4.152297184	3.962378139	4.203430041	4.151145462	3.978185501

180 days	A	3.860532523	4.208587947	4.256045786	4.084720819	4.254904531	4.317506874	4.061522956
	B	3.860532523	4.201136887	4.197696287	4.021973619	4.196549189	4.322046643	4.13327862
	C	3.79823223	4.077766587	4.176456144	4.049905639	4.209160903	4.309558025	4.000977445

270 days	A	3.776785136	4.294212764	4.366217491	4.137892149	4.392753571	4.442279551	4.158629545
	B	3.895376476	4.18392344	4.270871825	4.150569557	4.308422033	4.389933406	4.069647769
	C	3.891838301	4.323748602	4.357170323	4.137892149	4.358867196	4.365086974	4.164958342

365 days	A	3.948307546	4.393317523	4.434976112	4.21145244	4.348116202	4.510604955	4.195401974
	B	2.503436224	4.378646039	4.379775259	4.281124862	4.378646039	4.404590959	4.208014962
	C	4.012647003	4.350946363	4.446210333	4.168983907	4.421481136	4.503342676	4.194254644

The article "Performance Evaluation of Bio Concrete by Cluster and Regression Analysis for Environment Protection" was published in 2022. Journal: Comput Intell Neurosci.

## Data Availability

Data are available on request.
